# IoT Workflow Scheduling Using Intelligent Arithmetic Optimization Algorithm in Fog Computing

**DOI:** 10.1155/2021/9114113

**Published:** 2021-12-24

**Authors:** Mohamed Abd Elaziz, Laith Abualigah, Rehab Ali Ibrahim, Ibrahim Attiya

**Affiliations:** ^1^Department of Mathematics, Faculty of Science, Zagazig University, Zagazig 44519, Egypt; ^2^Academy of Scientific Research and Technology (ASRT), 101 Qasr Al Aini St., Cairo PO Box 11516, Cairo, Egypt; ^3^Artificial Intelligence Research Center (AIRC), Ajman University, Ajman 346, UAE; ^4^Faculty of Computer Science Engineering, Galala University, Suze 435611, Egypt; ^5^School of Computer Science and Robotics, Tomsk Polytechnic University, Tomsk 634050, Russia; ^6^Faculty of Computer Sciences and Informatics, Amman Arab University, Amman 11953, Jordan; ^7^School of Computer Sciences, Universiti Sains Malaysia, Gelugor, Pulau Pinang 11800, Malaysia

## Abstract

Instead of the cloud, the Internet of things (IoT) activities are offloaded into fog computing to boost the quality of services (QoSs) needed by many applications. However, the availability of continuous computing resources on fog computing servers is one of the restrictions for IoT applications since transmitting the large amount of data generated using IoT devices would create network traffic and cause an increase in computational overhead. Therefore, task scheduling is the main problem that needs to be solved efficiently. This study proposes an energy-aware model using an enhanced arithmetic optimization algorithm (AOA) method called AOAM, which addresses fog computing's job scheduling problem to maximize users' QoSs by maximizing the makespan measure. In the proposed AOAM, we enhanced the conventional AOA searchability using the marine predators algorithm (MPA) search operators to address the diversity of the used solutions and local optimum problems. The proposed AOAM is validated using several parameters, including various clients, data centers, hosts, virtual machines, tasks, and standard evaluation measures, including the energy and makespan. The obtained results are compared with other state-of-the-art methods; it showed that AOAM is promising and solved task scheduling effectively compared with the other comparative methods.

## 1. Introduction

The Internet of things (IoT) has recently become an attractive topic in network applications, which deal with various connection-based Internet devices [1, 2]. In IoT, popular intelligent tools, such as mobile devices, smartphones, pads, laptops, smart cars, and sensor nodes, are increased by employing different items, such as sensors, modern intelligent appliances, cameras, defense methods, smart watches, robots, and transports [3]. IoT's primary purpose is to offer different applications and services, for example, manufacturing, transportation, medical treatment, transfer instrument, energy management, health care, and industrialization. These IoT utilizations mainly generate an enormous volume of data that necessitate being processed, collected, stored, and analyzed to gain valuable reports to accomplish the user's demands and interests [4, 5]. The massive number of IoT applications' characteristics is proliferating and demanding a high processing capability and experience that even the standard smartest devices cannot currently coordinate [6, 7].

Cloud environments are considered a powerful platform to fortify and support IoT populations. Cloud computing (CC) is the on-demand availability of network machine resources, particularly storage and computing capability, without immediate effective control by the end user. CC is commonly utilized to define data centers possible to various users across the Internet [8]. Several limitations of modern smart things, such as storage capacity, battery continuance, network devices, home appliances, and treatment ability, can be determined by finding the optimal condition demand and executing specific jobs in strong computing ecosystems, such as fog and cloud computing, while additionally giving easy tasks for smart things to succeed. A recently distributed computing environment, fog computing (FC), promotes IoT ecosystems [9]. It is a heterogeneous computing paradigm composed of machines named the fog nodes, which encourages applications, maintains meaningful data, and distributes connection capacity. Recap fog computing is an updated cloud computing version by distributing intelligence devices based on exchangeable users [10, 11]. The scheduling approach is employed to produce high and cost-effectiveness over fog connections. Fog computing provides less response time and fewer transportation difficulties in the system [12], but this will produce additional difficulties for task scheduling and resource allocation. These difficulties need to be addressed.

The fog computing is organized over a three-layer network as presented in Figure 1. The top layer is the cloud computing center region, typically covered by cloud computing collecting, warehousing, and preparing a vast amount of tasks. The middle fog-adding part generally is covered by fog nodes with particular computing energy and supports portability. The bottom layer is the IoT design region of users, which typically involved smartphones, laptops, cars, sensors, PC machines, etc. [13].

Task scheduling has an expanded distribution framework in cloud computing. Still, many things affect job efficiencies, such as varying loads and extreme usage of resources [14]. This process creates a long latency and weights out over the data center; therefore, the advent of FC is significant [15]. FC task scheduling is the prevalent underlying issue of changing the specifications and allocating resources [16]. There are several user specifications for IoT environments. Simultaneously, the FC device's service quality is slightly better than the cloud computing platform's service quality.

Effectively designating tasks in FC and designating them as per the users' requirements to ensure optimal scheduling are a big issue that needs to be handled. The multitask scheduling topic's time complexity is known to be NP-hard [1]; the literature has also recommended numerous intelligence optimization techniques [17, 18]. Li et al. [19] advanced a new resource scheduling approach by integrating the fuzzy clustering algorithm along with particle swarm optimization to improve user satisfaction in fog environments. In [20], Nguyen et al. suggested an optimization method for dealing with IoT devices in FC systems to address the work scheduling problem. To execute many tasks in the cloud-fog networks, the suggested approach's critical goal is to achieve an optimum balance between time cost and work arrangements. A novel workflow scheduling strategy focused on utilizing an enhanced variant of the ant colony algorithm in multiple processor ecosystems was proposed by Boveiri et al. in [21]. A new advanced algorithm was implemented by Tong et al. in [22] by integrating the power of the neural network and the Q-learning method, specifically the allocation of Q-learning tasks. In cloud computing technology, the suggested algorithm is aimed at solving IoT workflow scheduling.

Yang et al. in [23] introduced a new task allocation approach focused on utilizing the game technique to maximize the efficiency of the Internet objects activities in CC methods. A multi-objective optimization technique is suggested in [13] to address the job scheduling in FC ecosystems. In this analysis, a couple of principal variables are determined: the output rate and the allocation of resources. In [24], Mtshali et al. conducted a workflow scheduling scheme according to a visualization approach to create a helpful approach that can evaluate the optimum energy damage in fog computation circumstances with a low delay. A work scheduling method utilizing the moth-flame optimizer to determine a collection of jobs for FC nodes was proposed by Ghobaei-Arani et al. in [25]. This strategy aimed to achieve QoS satisfaction by minimizing the overall performance time of the tasks. A modern intelligent task scheduling approach utilizing a gray wolf optimizer to address CC challenges was suggested by Abualigah et al. in [16]. This approach aimed to find the optimum cost of time and resource distribution of the instrument's question. Zeng et al. in [26] proposed the job scheduling approach in FC ecosystems to support secured devices. The suggested approach has developed an optimized approach to schedule tasks and manage the resources with reduced task execution time to facilitate user operation.

Abdel-Basset et al. in [27] introduced a multi-objective strategy to address the task scheduling for multiprocessor systems using the adjusted sine-cosine optimizer. The proposed method optimizes the makespan and energy. The proposed method is analyzed with several common multi-objective methods: it obtained superior results in most of the test cases. Xueying Guo introduced a CC approach for scheduling based on using multi-objective optimization based on a self-defense mechanism [28]. Several factors are taken in this research including least time, load balance, and the cost function. The empirical results revealed that the proposed method enhanced the performance of the original method and obtained better scheduling results compared with other methods.

The general results of the task scheduling in the fog computing domain still need further investigation to obtain better results from the given studies. However, the latest developments can be better in regard to energy loss and makespan measures. Thus, we found a potential direction to investigate workflow scheduling in FC further. In the literature, it is also clear that the most suitable methods that have been successfully used in this domain are the modified and improved optimization methods. As observed, a new advanced approach using the improved technique is needed to solve the scheduling problems. The need of finding a new method to solve various task scheduling problems has become very important as this time the demands of the IoT applications in cloud computing become more and more.

In the same context, arithmetic optimization algorithm (AOA) is an evolutionary metaheuristic technique proposed by Abualigah et al. in [29]. Evolutionary algorithms proved their ability to address various real-world engineering problems [30], which motivated us to conduct this research using the recently introduced evolutionary optimization method (i.e., AOA). AOA employs the distribution behavior of the leading arithmetic operators in mathematical science, including multiplication (M), division (D), subtraction (S), and addition (A). This algorithm was recently successfully employed to address various complicated optimization problems, such as classical benchmark functions, advanced CEC2005 benchmark functions, and real-world engineering design problems. However, the performance of AOA still requires more improvement, especially during the exploitation phase. This motivated us to enhance the ability of AOA and apply it to real-world problems. In this research, an intelligent IoT application workflow scheduling method is proposed based on the use of the AOA in FC ecosystems, called AOAM. The suggested method improved the conventional AOA using effective and powerful operators from the MPA [31]. In general, MPA is a metaheuristic technique proposed to solve various engineering problems. It is inspired by the general foraging approach, namely Levy distribution and Brownian movements in ocean predators and optimal defiance rate method in biological communication between predator and prey.

AOA and MPA operatives' advantages are linked to achieve a robust method to tackle the task scheduling problems efficiently. The proposed approach seeks to optimize the total energy consumption and makespan time values experimented in this study to test IoT devices' QoS specifications. Comprehensive experiments with different datasets and task sizes validate the proposed AOAM performance. The achieved results demonstrate that the suggested AOAM gets more excellent results in almost all analysis scenarios. It is a powerful and promising task scheduling approach compared with other well-known comparative methods reported before.

The main improvements of this study are listed as follows:

- An intelligent hybrid workflow scheduling approach is proposed to utilize the arithmetic optimization algorithm (AOA) for IoT device utilization in fog computing environments
- We analyzed IoT devices' QoS demands in terms of total energy consumption and makespan measures
- We assessed the effectiveness of the developed AOAM system in terms of several different standard evaluation criteria by providing comprehensive experiments with different task utilization scenarios

This study's structure is rendered as follows: Section 2 presents the problem formulation and fitness function used to handle the task scheduling problem. Traditional arithmetic optimization algorithm and MPA are discussed in Section 3. The suggested IoT task scheduling using the enhanced optimization of AOA is given in Section 4. In Section 5, the experimental results and discussion are provided. In Section 6, we concluded the successes and proposed future work.

## 2. Model and Problem Description

This part explains the system design and the communication among various elements involved in the task scheduling phase of the suggested system. The task scheduling problem is then formulated.

### 2.1. System Model

This study assumes that the fog broker built in the fog layer is the main component of the suggested framework. The fog broker consists of three primary parts: task receiver, cloud-fog information duty, and task scheduler (TS). The task receiver gets all task demands obtained from IoT things and subscribers. This component manages the IoT tasks' characteristics and service requirements and then transmits them to the task scheduler. The cloud-fog information service gathers and monitors status reports of the resources possible. Also, it gives the computing nodes' status with the TS to better prepare proper schedule decisions. The TS deals with task scheduling by assigning the task requests to the relevant computing nodes following the task characteristics and the available resources' capabilities. Finally, handling the task applications is collected and returned to the fog mediator, which forwards them to the corresponding customers.

### 2.2. Problem Description

In this section, we introduce the mathematical description of the task scheduling problem. Consider there are *n* independent tasks (*T*={*T*_1_, *T*_2_, *T*_3_,…, *T*_*n*_}) that are received by the fog mediator to be passed through the CC and FC environments. These tasks have properties such as input/output file size, memory requirement, and task length (millions of instructions (MI)). In addition, assume that the system of cloud-fog contains a set of *m* computing nodes (CN) that consists of *m*_cloud_ and *m*_Fog_ nodes (i.e., CN=*m*_cloud_ ∪ *m*_Fog_). Each CN_*j*_,  *j*=1,2,…, *m* holds its characteristics such as storage capacity, memory size, network bandwidth, and CPU processing rate (millions of instructions per second (MIPS)).

Therefore, the expected computing time of *T*_*k*_,  *k*=1,2,…, *n* requests on CN_*j*_,  *j*=1,2,…, *m* is given by ECT and the task scheduler used it to determine the suitable schedule decision [32]. In general, the ECT of the task *T*_*k*_ on CN_*j*_ is represented by ECT_*k*,*j*_ and computed using the following equation:

(1) $$\begin{array}{c} {\text{ECT}}_{k,j}=\frac{{\text{TL}}_{k}}{P_{j}}. \end{array}$$

In equation (1), *P*_*j*_ denotes the processing speed of CN_*j*_ and TL_*k*_ denotes the length of task *T*_*k*_. The makespan (MK) computed for a schedule *X* is given as follows:

(2) $$\begin{array}{c} \text{MK}\left(X\right)=\underset{j\in 1,2,\ldots ,m}{\max}\sum_{k=1}^{n}{\text{ECT}}_{k,j}. \end{array}$$

The energy consumption of the server represents nearly 60% of its active state. The energy consumption of CN_*j*_ is represented by the energy consumed in its idle and active states. Also, the idle time of each CN_*j*_ is denoted by its execution time subtracted from its makespan. So, the energy consumption of CN_*j*_ (in terms of Joules) can be formulated as follows:

(3) $$\begin{array}{c} E\left({\text{CN}}_{j}\right)=\left(Et_{j}\times b_{j}+\left(\text{MK}-Et_{j}\right)\times a_{j}\right)\times P_{j}, \end{array}$$

(4) $$\begin{array}{c} b_{j}=10^{-8}\times P_{j}^{2}, \end{array}$$

(5) $$\begin{array}{c} a_{j}=0.6\times b_{j}. \end{array}$$

In equation (3), Et_*j*_ and MK represent the total execution time and makespan of CN_*j*_. *b*_*j*_ denotes the consumed energy in the active state for CN_*j*_. The total energy consumption (Tot_eng_) in cloud-fog environment can be calculated as follows:

(6) $$\begin{array}{c} {\text{Tot}}_{\text{eng}}=\sum_{j=1}^{m}E\left({\text{CN}}_{j}\right). \end{array}$$

### 2.3. Fitness Function

In this portion, the formulation of the fitness function used to determine the solution's quality for the task scheduling problem is given. Our objective is to optimize the makespan and total energy consumption since both have major influence on the overall performance of the fog system. This problem is considered a bi-objective problem, and the fitness function can be formalized as follows:

(7) $$\begin{array}{c} \text{Fit}=\eta \times {\text{Tot}}_{\text{eng}}+\left(1-\eta \right)\times \text{MK,} \end{array}$$

where *η* denotes the balance parameter between the two factors of the fitness function. Hence, our task scheduling objective is to minimize Fit. In general, the weighted sum approach is used to solve the current bi-objective optimization problem (i.e., makespan and total energy consumption). This approach has high ability to determine a single unique solution for the tested problem. Followed [33, 34], the minimization of equation (7) is always Pareto optimal.

## 3. Algorithm Background

### 3.1. Arithmetic Optimization Algorithm (AOA)

Within this section, the mathematical inspiration of arithmetic optimization algorithm (AOA) [29] as metaheuristic techniques is introduced. In general, AOA emulates the function of the basic arithmetic operators (i.e., subtraction *S*, addition (*A*), division (*D*), and multiplication (*M*)).

AOA starts with building the initial candidate solutions (*X*), which consists of *N* solutions, as given in

(8) $$\begin{array}{c} X=\left[\begin{array}{ccccc} x_{1,1} & \cdots & x_{1,j} & x_{1,n-1} & x_{1,n}\\ x_{2,1} & \cdots & x_{2,j} & \cdots & x_{2,n}\\ \vdots & \vdots & \vdots & \vdots & \vdots \\ x_{N-1,1} & \cdots & x_{N-1,j} & \cdots & x_{N-1,n}\\ x_{N,1} & \cdots & x_{N,j} & x_{N,n-1} & x_{N,n} \end{array}\right], \end{array}$$

where *n* represents each solution's dimension, and then, AOA computes the fitness value of *X*_*i*_,  *i*=1,2 …, *N* and finds the best solution *X*_*b*_. Then, the solutions (*X*) are updated according to either the exploitation phase or the exploration phase, and this is determined based on the value of the math optimizer accelerated (MOA) function formulated as follows:

(9) $$\begin{array}{c} \text{MOA}\left(t\right)={\text{Min}}_{M}+t\times \left(\frac{{\text{Max}}_{M}-{\text{Min}}_{M}}{t_{\max}}\right), \end{array}$$

where *t* denotes the current iteration, and Max_*M*_ and Min_*M*_ refer to the accelerated function's maximum and minimum values, respectively.

In the exploration phase, the updating process is performed using the division (*D*) or multiplication (*M*) operators. Followed [29], these operators are used to explore the search space to discover the infeasible region. The mathematical formulation of updating each solution (*X*_*i*_,  *i*=1,2,…, *N*) in the current population *X*, based on the current best solution *X*_*b*_ at iteration *t*, is given as follows:

(10) $$\begin{array}{c} X_{i,j}\left(t+1\right)=\left\{\begin{array}{c} \frac{X_{b,j}}{\left(\text{MOP}+\varepsilon \right)}\times \left(Dm_{j}+{\text{LB}}_{j}\right),\;\text{if }r2<0.5,\\ X_{b,j}\times \text{MOP}\times \left(Dm_{j}+{\text{LB}}_{j}\right),\;\text{otherwise.} \end{array}\right. \end{array}$$

In equation (10), Dm_*j*_=*D*_*j*_ × *μ*UB*j* and LB*j* are boundaries of search space at *j*th dimension. *D*_*j*_=(UB_*j*_ − LB_*j*_), and *ε* is very small number to avoid division by zero. *μ*=0.5 refers to a control parameter value, whereas MOP denotes the probability of the math optimizer, which is formulated as follows:

(11) $$\begin{array}{c} \text{MOP}\left(t\right)=1-\frac{t^{1/\alpha }}{t_{\max^{1/\alpha }}}. \end{array}$$

In equation (11), *t*_max_ signifies the maximum number of iterations. *α*=5 is a dynamic parameter used to specify the precision of exploitation search method.

Moreover, in the exploitation phase, the addition (*A*) and subtraction (*S*) are used to update the solutions (*X*) inside the discovered feasible region. The formulation of this updating process is given as follows:

(12) $$\begin{array}{c} X_{i,j}\left(t+1\right)=\left\{\begin{array}{cc} X_{b,j}-\text{MOP}\times \left(D_{j}\times \mu +LB_{j}\right), & r3<0.5,\\ X_{b,j}+\text{MOP}\times \left(D_{j}\times \mu +LB_{j}\right), & \text{otherwise.} \end{array}\right. \end{array}$$

In equation (12), *r*3 ∈ [0,1] refers to a random number applied to control the process of using either the subtraction operator or the addition operator.

Thereafter, the updating process of the solutions is repeated until reaching the stop conditions and then returning the best solution *X*_*b*_. The details of AOA are outlined in Algorithm 1.

### 3.2. Marine Predators Algorithm

This section introduces the steps of the marine predators algorithm (MPA) [31]. In general, MPA emulates the behavior of predators to catch the prey. The first step in MPA is to produce a set of *N* solutions *X* using the following equation:

(13) $$\begin{array}{c} X=\text{LB}+\text{rand}\times \left(\text{UB}-\text{LB}\right), \end{array}$$

where rand ∈ [0,1] denotes a random number. LB and UB are the limit boundaries of search space [35]. Then, the Elite matrix is constructed as formulated in the following equation:

(14) $$\begin{array}{c} \text{Elite}=\left[\begin{array}{cccc} X_{11}^{1} & X_{12}^{1} & \ldots & X_{1\;d}^{1}\\ X_{21}^{1} & X_{22}^{1} & \ldots & X_{2\;d}^{1}\\ \ldots & \ldots & \ldots & \ldots \\ X_{n1}^{1} & X_{n2}^{1} & \ldots & X_{n\;d}^{1} \end{array}\right]. \end{array}$$

The process of updating the solutions is performed through three stages [36], and the details of these stages are given as follows:

(1) In the first stage, the prey is faster than the predator. So, the predator still moves without stopping and this happens during the first third of the optimization period. The mathematical formulation of updating the position of prey is given as follows:
  (15) $$\begin{array}{c} S_{i}=R_{B}\times \left({\text{Elite}}_{i}-R_{B}\times X_{i}\right),\;i=1,2,\ldots ,N, \end{array}$$
  (16) $$\begin{array}{c} X_{i}=X_{i}+P\times R\times S_{i},\;P=0.5. \end{array}$$
In equation (16), *R* ∈ [0,1] denotes a random number and *R*_*B*_ represents a Brownian motion value.
(2) In the second stage, it is considered that the prey and the predator have the same velocity. This happens during the middle interval of the period. The predator and prey's movement is simulated using the Brownian technique and the Levy flight technique, respectively. Within this stage, *X* is divided into halves; the first half is updated using the following equations:
  (17) $$\begin{array}{c} X_{i}=X_{i}+P\times R\times S_{i}, \end{array}$$
  (18) $$\begin{array}{c} S_{i}=R_{L}\times \left({\text{Elite}}_{i}-R_{L}\times X_{i}\right),\;i=1,2,\ldots ,N. \end{array}$$
In equation (17), *R*_*L*_ denotes the value generated using Levy distribution. Meanwhile, the second half of *X* is updated using the following equation:
  (19) $$\begin{array}{c} X_{i}={\text{Elite}}_{i}+P\times \text{CF}\times S_{i}, \end{array}$$
  (20) $$\begin{array}{c} \text{CF}={\left(1-\frac{t}{t_{\max}}\right)}^{\left(2t/t_{\max}\right)}, \end{array}$$
  (21) $$\begin{array}{c} S_{i}=R_{B}\times \left(R_{B}\times {\text{Elite}}_{i}-X_{i}\right),\;i=1,2,\ldots ,N, \end{array}$$
   where *t* and *t*_max_ are the present and maximum number of iterations, respectively.
(3) In the third stage, it is considered that the predator has velocity faster than the velocity of the prey, and this occurred during the last third of the optimization period. The mathematical formulation of updating the solution is given in the following equation:

(22) $$\begin{array}{c} X_{i}={\text{Elite}}_{i}+P\times \text{CF}\times S_{i}, \end{array}$$

(23) $$\begin{array}{c} S_{i}=R_{L}\times \left(R_{L}\times {\text{Elite}}_{i}-X_{i}\right),\;i=1,2,\ldots ,N. \end{array}$$

Followed [31], the eddy formation and fish aggregating devices (FADS) can change the behavior of the predators, and MPA formulated this as in the following equation:

(24) $$\begin{array}{c} X_{i}=\left\{\begin{array}{cc} X_{i}+\text{CF}\left[\text{LB}+R\times \left(\text{UB}-\text{LB}\right)\right]\times U, & r_{5}<\text{FAD},\\ X_{i}+\left[\text{FAD}\left(1-r\right)+r\right]\left(X_{r1}-X_{r2}\right), & r_{5}>\text{FAD}. \end{array}\right. \end{array}$$

In equation (24), *U* refers to a binary vector, FAD=0.2; *r*, *r*_1_, and *r*_2_ are random values in [0, 1].

In addition, a marine has a memory that supports its ability to remember its previous position. So, this behavior is added to the MPA by comparing the current position with its previous one. The full steps of MPA are given in Algorithm 2.

## 4. The Proposed Task Scheduler

Within this section, the main steps of the developed task scheduler method are introduced as in Figure 2. This proposed method depends on improving the arithmetic optimization algorithm (AOA) behavior using the advantages of MPA. The main target of using MPA is to enhance the local searching ability of AOA. This leads to avoid attraction to local points and increase the convergence speed.

The first step of the developed task scheduler method, named AOAM, is to construct the initial population *X*, which contains *N* solutions. Then, the fitness value (Fit_*i*_) is calculated and the best solution (*X*_*b*_) is determined. Thereafter, the solutions *X* inside the current population are updated using AOA and MPA operators. This process of updating solutions is repeated until the terminal conditions are satisfied and return *X*_*b*_. The description of the developed method is given in the following sections with more details.

### 4.1. Initial Phase

In this phase, the initial population *X* is constructed using the following equation:

(25) $$\begin{array}{c} X_{ij}=\text{floor}\left({\text{LB}}_{ij}+\text{rand}\times \left({\text{UB}}_{ij}-{\text{LB}}_{ij}\right)\right),\;j=1,2,\ldots ,n. \end{array}$$

In equation (25), rand ∈ [0,1] is a random number. LB and UB refer to the limitations of the search space, and it is set to 1, and *N*_*M*_ denotes the number of computing nodes. The dimension of *X*_*i*_ is set to *N*_*T*_, representing the number of tasks. floor(·) is applied to convert the actual values to discrete values. This is suitable for this kind of discrete optimization problem, such as task scheduling problems.

### 4.2. Updating Stage

In this phase, AOAM determines the quality of each solution by computing its fitness value (Fit_*i*_) that is given in equation (7), followed by determining the smallest fitness value and its corresponding solution, which represents the best solution *X*_*b*_. The next step is to adopt the current population *X* using AOA and MPA operators as given in the following equation:

(26) $$\begin{array}{c} X_{i}\left(t+1\right)=\left\{\begin{array}{cc} \text{update }X_{i}\text{ using AOA} & \text{if rand}\geq 0.5,\\ \text{update }X_{i}\text{ using MPA} & \text{if rand}<0.5, \end{array}\right. \end{array}$$

where rand ∈ [0,1] is a random number used to switch between AOA and MPA operators.

Finally, the stop conditions are checked, and when they are satisfied, the steps of the updating phase are stopped and the best solution *X*_*b*_ is returned. The pseudo-code of the AOAM is given in Algorithm 3.

### 4.3. Computational Complexity Analysis

This subsection provides the time complexity analysis of the aforementioned three algorithms. Assume *N* be the population size (number of solutions), *M* is the number of iterations, and *L* is the number of parameters (dimension). The computational complexity of AOA is *O*(*N* × (*M* × *L*+1)) [29]. The computational complexity of MPA is *O*(*M* × (*N* × *L*+Cof*∗N*)) [31], where Cof signifies the objective function cost. According to the steps of the proposed AOAM algorithm, the time complexity of population initialization (step 2 of the algorithm) is *O*(*N*) and the time complexity of updating solutions (steps 4 − 11 of the algorithm) is *O*(*N* × *M*). Therefore, the overall time complexity of AOAM is *O*(*N*+*N* × *M*), that is, *O*(*N* × *M*).

## 5. Experimental Studies

This section offers a detailed experimental performance evaluation of the contributions suggested in this study. In particular, the simulation settings and datasets are introduced in Section 5.1. The performance metrics are described in Section 5.2. Finally, the experimental results along with discussions are provided in Section 5.3.

### 5.1. Experimental Settings

All the experiments are conducted using MATLAB R2018a on a Dell PC configured with an Intel Core i5 CPU of 2.40 GHz frequency, 4GB RAM, and Windows 10 operating system. We remark the MATLAB simulator's widespread adoption for evaluating the schemes published in the literature [37–39]. The cloud-fog framework in our tests consists of fog nodes that have small processing power. However, they are closer to the IoT devices and have a minimal delay. On the other hand, cloud nodes can quickly execute IoT tasks, but they need a long time to embrace them. The FC ecosystem contains two data centers, 4 hostess machines, and 20 VMs of various arrangements in all of the tests.

Consequently, the suggested algorithms should manage the equilibrium between fog and cloud nodes to enhance system performance.  Table 1 lists the attributes of the hosts and VMs. As represented in Table 1, the most inactive and active VM processing capacities are 1000 and 5000 MIPS, respectively.

In our experiments, both synthetic and natural workloads are mainly involved. The real workloads are generated from the “Parallel Workload Archives” that consist of HPC2N and NASA Ames iPSC/860. These workload archives are made available to the research community in the standardized workload format (SWF) [40]. The NASA iPSC log comprises about 42,264 tasks, while the HPC2N comprises about 527,371 tasks. On the other hand, the synthetic workload consists of 1500 tasks with lengths ranging from 2,000 to 56,000 MI generated from a uniform distribution. The specification of the synthetic workload is listed in Table 2.

### 5.2. Evaluation Metrics

In this article, our objective is to guarantee lower energy consumption with a better makespan. We measured the overall energy consumption and makespan for assessing the efficiency of the AOAM against other peer algorithms. In the following, we present those two performance metrics.

The makespan is defined as the completion time of the last accomplished task. A minimum makespan implies efficient mapping of user tasks to CN*s*. Makespan is computed on the basis of equation (2).

The total energy consumption is defined as the energy consumed by the physical resources (which involves all cloud and fog nodes). For a practical system, the energy consumption of the CN*s* should be minimal. The total energy is calculated as specified in equation (6).

### 5.3. Results and Discussion

For comparative analysis, five state-of-the-art algorithms, including the standard AOA [29], Manta ray foraging optimization (MRFO) algorithm [41], marine predators algorithm (MPA) [31], Chimp optimization algorithm (CHOA) [42], Salp swarm algorithm (SSA) [43], and AEOSSA [10], are chosen as peer algorithms in this study.  Table 3 lists the parameter settings for all peer algorithms. Each algorithm was independently performed 30 times on each test instance to achieve more accurate estimates of our results. To ensure a fair comparison, the population size for each algorithm is set to 100. Moreover, *η* is set to 0.7 since our main concern is to reduce energy consumption. The parameters of each algorithm are based on its original implementation.

To study the performance behavior of the proposed AOAM algorithm, we plotted curves for the average fitness values obtained by AOAM and other comparison algorithms (MRFO, MPA, AOA, AEOSSA, SSA, and CHOA) for a different number of tasks, as shown in Figures 3–5. The curves visualize the average fitness values generated by the algorithms for different datasets and task sizes. The number of tasks is shown along the *x*-axis. At the same time, the value of the fitness function is represented along the *y*-axis. Note that the fitness value is impacted by 70% of the total energy consumption value plus 30% of the value of the makespan.

The curve of the synthetic workload is illustrated in Figure 3. The figure shows that the AOAM algorithm succeeded in obtaining lower fitness values compared with other methods when tasks vary between 300 and 1500. Similarly, the curve of fitness values for NASA Ames iPSC dataset depicted in Figure 4 establishes the better performance of the AOAM algorithm as compared to other comparison algorithms. Moreover, AOAM has succeeded in attaining lower fitness values than other scheduling approaches for the HPC2N actual workload, while the tasks vary from 1000 to 5000, as seen in Figure 5. The curves present that combining the MPA method with the AOA boosts its ability to find near-optimal solutions.

Figures 6–8 present the average makespan results obtained by the AOAM, AOA, MRFO, AEOSSA, MPA, SSA, and CHOA for the synthetic and real datasets with different task sizes. From Figure 6, we see that the AOAM is significantly better than the other peer algorithms on all of the synthetic instances considered. Similarly, from Figure 7, we can see that the AOAM performs significantly better than all of the other peer algorithms across all NASA Ames iPSC instances. Moreover, we can see from Figure 8 that the AOAM is substantially better compared with other five peer methods over all the HPC2N scenarios. Finally, the figures' results indicate that AOAM generates the best makespan among all six peer algorithms for all the tested instances.

The comparison of the total energy consumption between AOAM, AOA, AEOSSA, MRFO, MPA, SSA, and CHOA using both synthetic and real workload traces is shown in Figures 9–11.  Figure 9 shows that the proposed AOAM algorithm attains the lowest energy consumption compared with the original AOA and other peer algorithms for the synthetic dataset. Similarly, Figure 10 shows that the proposed algorithm, AOAM, achieves the lowest energy consumption compared with the other peer algorithms when the NASA Ames iPSC workload is considered. Furthermore, Figure 11 illustrates that the AOAM provides the lowest energy consumption in contrast to other peer algorithms when the HPC2N workload is taken into account. In a nutshell, the comparison results reveal that AOAM generates a better energy consumption than all other peer algorithms for all task sizes and datasets.

### 5.4. Statistical Results

To assess whether there are significant improvements in the results obtained by the developed method and other methods, a nonparametric test named the Friedman test is used. This test provides a *P* value that indicates whether the control group (AOAM) has a significant difference with other MH techniques or not based on different performance measures including makespan, energy, and fitness value. The mean rank of each algorithm over the tested datasets in terms of performance metrics is given in Table 4. From the given results, it can be seen that in terms of makespan the developed method has the best mean rank overall the competitive algorithms with *P* value of 1.39*e* − 4, whereas in terms of energy, it can be observed that the developed AOAM achieves the first rank followed by MRFO and AOA in the second and third ranks, respectively, over the three datasets.

In summary, the findings revealed that the AOAM algorithm provides better solution quality and diversity, thus leading to near-optimum solutions. Overall, the results shown above justify the advantage of incorporating the MPA strategy along with the AOA. Therefore, integrating MPA with the AOA can effectively increase the search efficiency to achieve better solutions for all examined workload instances.

## 6. Conclusion

Task scheduling is among the significant challenges in cloud and fog computing environments because of the variability and dynamicity of the resources and the high volatility of service requests from cloud subscribers. This study proposed a hybrid algorithm that combines AOA with the marine predators algorithm (MPA) to find an appropriate solution for optimizing the fog task scheduling. The suggested AOAM approach is an attempt to enhance the solution goodness and convergence ratio of the original AOA. The performance of AOAM is evaluated and contrasted with the standard AOA and other four optimization algorithms, including MRFO, MPA, AEOSSA, SSA, and CHOA. The experimental results confirm the effectiveness of our AOAM approach in terms of makespan and total energy consumption. More specifically, the obtained results revealed that the AOAM is better than the original AOA and outperforms all comparative algorithms in all of the tested instances.

In future work, we plan to investigate the performance of the AOAM approach in large-scale computing environments with hundreds of servicing nodes, considering more objectives such as response time, transmission costs, reliability, and security to fulfill the growing customer needs. In addition, AOAM could be further improved and integrated with other optimization algorithms to tackle more optimization problems such as vehicle routing problems, job shop scheduling, quadratic assignment, and traveling salesman problem.

## Figures and Tables

**Figure 1:** Fog computing structure.

**Figure 2:** Developed AOAM.

**Figure 3:** Fitness value for the synthetic workload.

**Figure 4:** Fitness value for real workload NASA iPSC.

**Figure 5:** Fitness value for real workload HPC2N.

**Figure 6:** Average makespan for the synthetic workload.

**Figure 7:** Average makespan for real workload NASA iPSC.

**Figure 8:** Average makespan for real workload HPC2N.

**Figure 9:** Total energy consumption for the synthetic workload.

**Figure 10:** Total energy consumption for real workload NASA iPSC.

**Figure 11:** Total energy consumption for real workload HPC2N.

**Algorithm 1:** Steps of AOA.

**Algorithm 2:** Steps of MPA.

**Algorithm 3:** AOAM scheduler.

**Table 1:** Characteristics of experimental parameters.

Cloud Entity	Parameter	Value
Datacenter	No. of data centers	2
Client	No. of clients	100–200
Host	No. of hosts	4
	Storage capacity	2 TB
	RAM	20 GB
	Bandwidth capacity	10 Gb/s
	Policy type	Time shared

VM	No. of VMs	20
	CPU power	1000–5000 MIPS
	RAM	2 GB
	Storage	10 GB
	Bandwidth capacity	1 Gb/s
	No. of CPUs	1

**Table 2:** Characteristics of synthetic workload.

Parameter	Value
No. of tasks	300 to 1500
Length of the task	2000 to 56 000 MI
File size	400 to 600 MB
Output size	400 to 600 MB

**Table 3:** Parameter settings of AOAM and peer algorithms.

Algorithm	Parameter	Value
AOA	MOP_Max_	1
	MOP_Min_	0.2
	*α*	5
	*μ*	0.499

MPA	FAD*s*	0.2
	*P*	0.5

CHOA	*a*	[−1, 1]
	*f*	2⟶0

MRFO	*S*	2
	*r*_1_, *r*_2_, *r*_3_	[0, 1]

SSA	*c*_1_, *c*_2_, and *c*_3_	[0, 1]

AOAM	MOP_Max_	1
	MOP_Min_	0.2
	*α*	5
	*μ*	0.499
	FAD*s*	0.2
	*P*	0.5

**Table 4:** Results of the Friedman test.

		SSA	CHOA	MPA	MRFO	AOA	AOAM	*P* value
Makespan	Synthetic	6	5	4	3	2	1	1.39*e* − 04
	NASA	6	5	4	3	2	1	1.39*e* − 04
	HPC2N	6	5	4	3	2	1	1.39*e* − 04

Energy	Synthetic	5.8	5.2	4	2.2	2.8	1	2.09*e* − 04
	NASA	6	5	3.6	2.4	3	1	3.13*e* − 04
	HPC2N	6	5	3.6	2	3.4	1	1.88*e* − 04

Fitness	Synthetic	5.8	5.2	4	2.2	2.8	1	2.09*e* − 04
	NASA	6	5	3.6	2.4	3	1	3.13*e* − 04
	HPC2N	6	5	3.6	2	3.4	1	1.88*e* − 04

## Data Availability

The data used to support the findings of this study are available from the authors upon request.
